This article has been retracted.

# Put the control back in the control condition: are brown, pink, and white noise neutral control stimuli?

**DOI:** 10.3389/fnins.2025.1488682

**Published:** 2025-04-25

**Authors:** Ulvhild H. Færøvik, Kjetil Vikene, Karsten Specht

**Affiliations:** ^1^Department of Biological and Medical Psychology, Faculty of Psychology, University of Bergen, Bergen, Norway; ^2^Department of Radiology, Mohn Medical Imaging and Visualization Centre, Haukeland University Hospital, Bergen, Norway; ^3^Department of Education, Faculty of Humanities, Social Sciences and Education, UiT The Arctic University of Norway, Tromsø, Norway

**Keywords:** control stimuli, control condition, brown noise, pink noise, white noise, GEMS-9

## Abstract

**Introduction:**

What are good control stimuli for music perception research? Systematic evaluations of control suitability remain limited. We wanted to examine if control stimuli (brown, pink, white noise, and voice recordings) lead to different emotional ratings in themselves.

**Methods:**

Across two separate studies (n = 84, and 1280, respectively), participants assessed brown, pink, and white noise and voice recordings using a music-emotional perception scale with variations. We used the GEMS-9 scale, and the GEMS-9 scale with the second-order factors ‘sublime’, ‘uneasy’, and ‘vital’.

**Results:**

Our two studies show that brown noise was considered more sublime than white and pink noise, while white noise was considered more uneasy than brown noise, pink noise, and voice recordings in both studies.

**Discussion:**

Brown, pink, and white noise is rated emotionally above 3 on unease on a scale from 1 to 7. This means that none of the noise stimuli had minimal emotional ratings and therefore had an emotional effect in themselves. Out of the three noise stimuli, white noise had the highest ratings of unease across both studies. Only voice recordings were considered neutral, defined as having consistently minimal emotional ratings in both studies.

## Introduction

The common incorporation of control conditions in experimental science dates to 1908 (Boring, 1954). Control conditions constitute an integral aspect of a research design, serving as essential comparators to experimental conditions and providing a reference point for evaluating the effects of independent variables (Pelham and Blanton, 2018). While not all studies include a control condition/stimuli, its inclusion is essential for the unbiased, objective observation for discerning effects beyond those attributed to the independent variable (Torday and Baluška, 2019).

Controlling control stimuli was the focus of the present article in the context of studies on music perception. Perhaps the best-known example of the importance of using control stimuli in studies on music is the “Mozart study” (Rauscher et al., 1993). In 1993, Raucher and coworkers showed that participants did better on an abstract spatial reasoning test when listening to music by Mozart compared to those who sat in silence or heard a relaxation tape. The “Mozart effect” was not found in subsequent replications (Carstens et al., 1995; Newman et al., 1995; Roth and Smith, 2008; Steele et al., 1997, 1999; Stough et al., 1994). Despite this example, not using appropriate control stimuli in studies with music has been noted as a prevailing issue (Chanda and Levitin, 2013; Koelsch and Jäncke, 2015).

To improve the prevailing issue Koelsch and Jäncke advocate for acoustical control stimuli, emphasizing their importance in contrasting with music conditions (2015). Conversely, Chanda and Levitin posit that control stimuli should be non-musical, highlighting the inconsistency of the optimal choice of control conditions in music-related research (2013). Others have suggested that familiar music should be compared to control conditions, such as silence and unfamiliar music (Hunt and Legge, 2015). However, silence as a control condition could increase the potential for a placebo effect, particularly when other conditions have an auditory component (Mallik and Russo, 2022). Groarke et al. (2020) underscore the importance of an active control condition in their two studies: one using silence and the other a radio show as a control condition. They observed an effect of music in the first study but not in the second, leading to a discussion on the impact of active versus passive control conditions (Groarke et al., 2020).

A passive control stimulus is something that does not require much attention from the participant, such as silence. An active control stimulus is something that requires attention from the participant, such as giving a subjective or physiological response. While researchers often try to use a “neutral” stimulus as a control condition, the stimuli have typically not been validated beforehand, which may lead to biases and false conclusions (Hahn et al., 2024). A control stimulus which has been frequently used in white noise.

White noise has been used in early neuroscience studies with cats (Galin, 1964; Starr and Livingston, 1963). Galin (1964) used tonal stimuli in comparison to white noise. Using tonal stimuli and white noise was done with human subjects shortly after (Bregman, 1978; Davis et al., 1968; Graham and Slaby, 1973). White noise has continued to be employed as a control stimulus in contrast to music (Bigliassi et al., 2015; Lynar et al., 2017; Nyklíček et al., 1997; Ozkalayci et al., 2016; Russo et al., 2013; Shokhadze, 2007). White noise is a sound containing all frequencies with equal intensities at all frequencies, which resembles the sound of ocean waves or wind (Aksoy and Ozturk, 2024) or a strong waterfall (Azizi and Yazdi, 2019).

White noise has previously been intended as a “neutral” stimuli baseline for heart rate compared to music (Lynar et al., 2017). However, a five-minute white noise session was associated with higher heart rate variability values and moderate relaxation ratings compared to three music conditions (high arousal jazz, low arousal classical, and participants choosing their uplifting music). This led the authors to conclude that “white noise was not effective as a neutral stimulus” (Lynar et al., 2017). Furthermore, white noise has been reported as unpleasant compared to pure tone stimuli, which consist of only single-frequency sounds with consistent intensity (Masuda et al., 2018). In addition, white noise control conditions have been reported to be less pleasant than different music and silence conditions (Bishop et al., 2009). Compared to classical music, white noise impaired cognitive functions during measures of conflict processing (Pascoe et al., 2022). Perhaps surprisingly, Justel et al. (2023) found that white noise enhanced recall compared to listening to music on a memory test in their initial study. However, in the subsequent study, music enhanced recall compared to white noise (Justel et al., 2023).

In the field of medicine, it has been reported that patients required less anesthesia when listening to music compared to white noise, although there was no difference in anxiety levels (Ayoub et al., 2005). However, nursing students felt more anxious when performing tasks with white noise in the background, as opposed to silence and music (Aksoy and Ozturk, 2024). Surprisingly, music was as inefficient as white noise and silence on sedation depths on dental procedures with children (Ozkalayci et al., 2016).

Taken together, the previous research on white noise seems to indicate that it is not a “neutral” control condition, which has not been thoroughly studied separately. It is worth nothing that some studies on music perception have not reported separate analyses specifically dedicated to the white noise used (Bigliassi et al., 2015; Loui et al., 2012; Russo et al., 2013; Shoda et al., 2016). Other control stimuli used with music are pink noise (which exhibits equal energy per octave, featuring more low-frequency components compared to white noise) and brown noise (which changes in frequencies at random).

Pink noise is distinguished from other noises that have a reddened spectrum, as the frequency variance continues to increase, no matter how long the time series is (Halley, 1996). Pink noise has been found to enhance sleep stability compared to silence (Zhou et al., 2012). Additionally, pink noise has been rated as quiet compared to classical music (Kreutz et al., 2003). Interestingly, traditional Chinese music led to an increase in functional connectivity in the alpha2 band, compared to both pink noise and silence conditions (Wu et al., 2013). Furthermore, music is better at reducing somatic anxiety compared to pink noise (Mallik and Russo, 2022). In a physiological study where pink noise served as the designated control condition, the authors did not report a separate pink noise analysis (Shoda et al., 2016). This highlights the distinct impact of different auditory stimuli on neural responses, however, there is little literature on pink noise compared to music.

Unlike white noise, brown noise decreases in power as the frequency increases (Azizi and Yazdi, 2019). Brown noise is sometimes referred to as red noise because it is somewhat analogous to a red light, which has a low frequency. Brown noise has been utilized as a neutral control to music (Moghimi et al., 2012). Interestingly, brown noise has been rated as more pleasant than white noise (Voss and Clarke, 1978). In addition, brown noise, brown noise together with binaural beats, brown noise and music, and all three conditions combined have been used to induce relaxation (Krasnoff and Chevalier, 2023). Moreover, pink and white noise is preferable as an additive noise to the amplitude-modulated tones to increase neural responses. Interestingly, brown noise does not exhibit the same efficacy in this context (Monobe et al., 2019). As with pink noise, there is little literature on brown noise compared to music.

Other control stimuli can be movies, music, and spoken and written stories, which tend to be rated with strong emotions and have ecological validity within a laboratory setting (Saarimäki, 2021). Some studies use voice recordings, such as audiobooks, to control for an effect compared to music (Jespersen et al., 2015; Sihvonen et al., 2020). As with brown and pink noise, voice recordings have not been frequently cited in the literature as a control stimulus to music.

The influence of brown, pink, and white noise on emotional responses has demonstrated various responses, prompting a need for further investigation, also in the context of the perception of music. Given the uncertainty surrounding appropriate control conditions, our research tries to address this gap through two studies utilizing the Genova Emotional Music Scale-9 (GEMS-9) (Zentner et al., 2008). The GEMS-9 consists of nine emotional labels, or first-order factors. The second-order factors are sublime, vital, and uneasy and encompass the first-order factors (Zentner et al., 2008).

### Aim and hypothesis

In this study, we aimed to explore the possibility of using brown, pink, and white noise as control stimuli, as well as voice recordings, based on the premise that they are rated with minimal emotional responses. We do not assume that the stimuli are strictly “neutral.” However, neutral stimuli have been defined as stimuli that people are indifferent to and lead to no preference (Gasper et al., 2019). Additionally, it has been shown that participants report feeling neutral alongside both positive and negative affect (Gasper et al., 2021), indicating that neutrality is a complex phenomenon perhaps not entirely devoid of emotion. Neutrality for our studies is defined as low ratings (below 3 out of 7), which were interpreted as either minimal emotional impact or the absence of emotion.

We anticipated that white noise would be rated with the strongest feelings of unease compared to brown noise, pink noise, and voice recordings. This is also somewhat consistent with previous literature where white noise was rated as unpleasant compared to music (Bishop et al., 2009; Lynar et al., 2017; Masuda et al., 2018). White noise has also been shown to be more unpleasant than pink noise (Voss and Clarke, 1978). We also assumed that noise stimuli and voice recordings would give minimal emotional responses (below 3, on a scale from 1 to 7).

## Methods

The two studies adopted a common methodological approach, utilizing a version of the GEMS-9 (Zentner et al., 2008). This scale, initially developed for the emotional validation of classical music, underwent a translation to Norwegian in 2014 at our department (See Supplementary Table 1 for translation and emotional words). We chose to use this scale as the music data in study 2 was part of a study on the emotional perception of music, and we wanted to be able to compare studies 1 and 2.

Volunteer participants across all studies were recruited through convenience and snowball sampling from the Norwegian-speaking population. The studies were conducted using an internet survey based on l.a.m.p. (Linux/Apache/MySQL/PhP) and HTML/Javascript/CSS, which we developed.

All procedures were approved by the Regional Committee for Medical and Health Research Ethics (REK 45655-2019) and carried out according to the Code of Ethics of the World Medical Association, Declaration of Helsinki. Electronic informed consent was obtained from all participants upon enrollment.

### Stimuli

Brown, pink, and white noise stimuli were sourced from YouTube for their availability and ease of access. All noises were subjected to a standardized editing procedure using Logic Pro X for Mac (Cousins and Hepworth-Sawyer, 2024). Each noise was adjusted to have a consistent duration of 21 s. As the current studies were part of a larger project on the emotional perception of music, stimuli length needed to be the same across controls and music. The duration was based on a review (Warrenburg, 2020) which found that 50% of music stimuli in emotion research fall under 30 s.

Both our studies were online surveys. Although the loudness of all stimuli was normalized, participants could adjust the volume of the stimuli. Spectral frequency power analyses were performed in MATLAB_R2021a on the three noises see Figure 1.

**Figure 1:** Displays the spectral frequency power analyses for all three noise stimuli; the black line represents white noise, the red line represents pink noise, and the blue line represents brown noise.

In addition, three voice recordings were selected as a control for the noise stimuli. The texts were two parts from a toaster instruction manual and one part from a boat ticket disclaimer. The voice recordings were read by both a male and a female reader with an East Norwegian accent. This dialect was used as it holds cultural dominance and therefore influences Norwegian culture (Papazian, 2012). Voice recordings were also recorded and edited with Logic Pro X for Mac (Cousins and Hepworth-Sawyer, 2024) and had a duration of 21 s. In total, six “neutral” non-emotional topic voice recordings were presented in the survey, and three texts were read by both a female and male reader (3×2 = 6).

All stimuli were normalized using Audacity (GNU General Public License, 2024). Normalizations were verified and measured with Brüel & Kjær Head and Torso simulator, type 2128C.^1^

In study 2, a diverse set of stimuli was employed, including 40 musical items (comprising songs with different tempi at 60, 100, 120, and 150, in both minor and major modes), white, pink, and brown noises, and 6 neutral speech stimuli were used. The analysis of stimuli other than the noise stimuli will be reported and published elsewhere and is not included in this paper.

### Participants

In study 1, volunteers (*N* = 84, 38 females, 45 males) were aged 18–77 years (mean age 32.3, SD =12.2). Most participants were right-handed (75). Educational background varied, with two participants not having completed basic education, 18 having completed basic education, 39 participants having some higher education, and 25 participants holding a master’s degree or a Ph.D.

In study 2 (*N* = 1,280, 757 females, 496 males), twenty-seven participants did not fill out any of the demographic information but were still included in the analysis. The age range spanned from 19 to 94 years, with a mean age of 40 (SD = 15.6). Most participants were right-handed (*N* = 1,086) followed by left-handed (*N* = 119), and 36 individuals identified as ambidextrous. Educational background varied, with one participant not having completed basic education, 22 participants having completed basic education, 218 participants having completed high school, 573 having some higher education, and 442 participants holding a master’s degree or a Ph.D.

## Study 1

### Procedure

The GEMS-9 scale with the full Likert scale ranging from 1 to 7 was employed for emotional rating. Participants were asked to rate sounds on nine different emotions.

Participants received a link, individual passwords, and usernames to access the survey. They were explicitly instructed to wear headphones, although this was not verified or tested by us. The 17 acoustical stimuli were presented in a randomized order, and participants used a 7-Likert scale, ranging from 1 (not at all) to 7 (very much), to rate emotions. Participants had the flexibility to advance to the next stimuli as soon as they had rated the sound on all nine emotions, allowing them the option to not necessarily listen to the full 21 s. The survey design allowed participants the freedom to play each stimulus multiple times if desired. The entire survey process took approximately 10 min.

### Analysis

We hypothesized that white noise would yield stronger ratings for uneasy factors (tension and sadness) compared to brown and pink noise and voice recordings. Yet, we also assumed that the noises would not be normally distributed with minimal emotional ratings. To test our second hypothesis, we conducted a Shapiro–Wilk normality test for our 9 control stimuli (brown, pink, white noise, three voice recordings female and male versions). The test revealed that none of the control stimuli had normal data distribution with a significant rating of <0.001. See Supplementary Table 2 for details.

As the data was not normally distributed, we used the Friedman test for each of the second-order factors, then followed up with a post-hoc test using Wilcoxon signed rank. These are non-parametric tests to compare the voice recordings and noises against each other. Non-parametric methods do not rely on assumptions about the underlying data distribution (Pallant, 2020).

Prior research with the GEMS-9 (Pearce and Halpern, 2015; Zentner et al., 2008) suggests using the second-order factors, which encompass the first-order factors: sublime (wonder, transcendence, tenderness, nostalgia, and peacefulness), uneasy (sadness and tension), and vitality (joyful activation and power). We decided to analyze the stimuli by combining first-order factors for the second-order factor sublime and similarly for the other two second-order factors, uneasy and vital.

Finally, we created a combined neutral voice recording stimuli, combining the three “neutral” texts with both female and male voices and the second-order factors. Leaving us with four sublime stimuli, four vital stimuli, and four uneasy stimuli. Bonferroni adjustments were set for the Wilcoxon signed-rank tests. The alpha (*α*) was changed based on the number of comparisons (6). 0.05/6 = 0.0083.

### Power

Using G*Power (Faul et al., 2007, 2009) version 3.1, the alpha error probability was set to 0.05 with a power of 0.95, and the required effect size for the Wilcoxon signed rank test was 0.3.

### Results

#### Sublimity

The Friedman test indicated a statistically significant difference in sublimity ratings for brown, pink, and white noise, and voice recordings *X*^2^ (3, *n* = 82) = 57.8, *p* < 0.001. A Wilcoxon Signed Rank Test was used to compare brown, pink, and white noise, and voice recordings on sublimity Brown noise was rated significantly higher on sublimity than white noise and voice recordings. A statistically significant difference emerged between pink and white noise on the ratings of sublimity, as well as voice recordings (see Table 1 for details).

**Table 1:** Wilcoxon signed-rank test, for sublimity ratings.

Emotion	Paired stimuli	Median	*z*	*N*	Sig (two-tailed)	*r*
Sublime	Brown Noise- White noise	2 1	−5.92	82	0.001	0.6
	Brown Noise- Voices recordings	2 1.2	−5.26	82	0.001	0.5
	Pink noise- White noise	1.8 1	−5.37	82	0.001	0.5
	Pink noise- Voice recordings	1.8 1.2	−4.13	82	0.001	0.4

#### Unease

The results of a Friedman test indicated that there was a statistically significant difference in unease ratings for brown, pink, and white noise, and voice recordings *X*^2^ (3, *n* = 82) = 63.9, *p* < 0.001. A Wilcoxon Signed Rank Test compared brown, pink, and white noise, and voice recordings on unease. White noise was rated significantly higher on unease compared to brown noise, pink noise, and neutral voice recordings. Pink noise was rated significantly higher for unease compared to brown noise and neutral voice recordings (see Table 2 for details).

**Table 2:** Wilcoxon signed-rank test, for unease ratings.

Emotion	Paired Stimuli	Median	*z*	*N*	Sig (two-tailed)	*r*
Unease	White noise- Brown noise	3 1.5	−6.59	82	0.001	0.7
	White noise- Pink noise	3 2	−3.28	82	0.001	0.3
	White noise- Voice recordings	3 1.7	−5.88	82	0.001	0.6
	Pink noise- Brown noise	2 1.5	−5	82	0.001	0.5
	Pink noise Voice recordings	2 1.7	−3.11	82	0.002	0.3

#### Vitality

The results of a Friedman test indicated that there was a statistically significant difference in vitality ratings for brown, pink, and white noise, and voice recordings *X*^2^ (3, *n* = 82) = 28.2, *p* < 0.001. A Wilcoxon Signed Rank Test was used to compare brown, pink, white noise, and voice recordings on vitality. There was a statistically significant difference between pink and brown noise and white noise, and voice recordings (see Table 3 for details). See Figure 2 for visual representation.

**Table 3:** Wilcoxon signed-rank test, for vitality ratings.

Emotion	Paired stimuli	Median	*z*	*N*	Sig (two-tailed)	*r*
Vitality	Pink noise- Brown noise	2 1.5	−3.13	82	0.002	0.3
	Pink noise White noise	2 1	−4.41	82	0.001	0.4
	Pink noise- Voice recordings	2 1.5	−4.35	82	0.001	0.4

**Figure 2:** Displays brown, pink, and white noise and the neutral voice recordings on the three second-order GEMS-9 factors: sublimity, unease, and vitality. The median value is displayed. The error bars show the interquartile intervals (25th and 75th).

#### Happy and sad news

The analysis of the happy and sad news articles is not included. Both the happy and the sad news audio recordings received minimal emotional ratings (below three out of seven) and, therefore, were not considered emotional stimuli. We choose to omit this analysis due to space constraints; raw data can be obtained upon request from the first author.

## Study 2

### Hypothesis

Based on the results from Study 1, we adjusted our second hypothesis for Study 2.

Noise stimuli and voice recordings will be rated with minimal emotional responses (median below 3), except unease ratings for white noise.

### Procedure

Like study 1, except stimuli were presented in a semi-random order, using six different randomizations to ensure that the noises and audio recordings consistently followed four music stimuli. Participants, on average, spent 16 min and 44 s to complete the survey.

### Analysis

As with study 1 a Shapiro–Wilk normality test revealed that none of the control stimuli had normal data distribution with a significant rating of <0.001. See Supplementary Table 3 for details.

Like study 1, we opted to use a Friedman test and post-hoc Wilcoxon signed rank test, which is the non-parametric alternative to a t-test. The voice recordings were also combined into three stimuli for the three different emotions (sublimity, unease, and vitality). Bonferroni alpha corrections were the same, 0.008.

To compare the results from studies 1 and 2, we used a Mann–Whitney U test.

### Power

Using G*Power (Faul et al., 2007, 2009) version 3.1, the alpha error probability was set to 0.05 with a power of 0.95, and the required effect size for Wilcoxon signed rank test was 0.09.

Using G*Power with a Mann–Whitney U test comparing the groups in study 1 (*N* = 84) and study 2 (*N* = 1,280), with alpha error set to 0.05 and power of 0.95, the required effect size was 0.3.

### Results

#### Sublimity

The results of a Friedman test indicated that there was a statistically significant difference in sublimity ratings for brown, pink, and white noise, and voice recordings *X*^2^ (3, *n* = 1,267) = 333.9, *p* < 0.001. A Wilcoxon signed rank test revealed a statistically significant difference between all six pairs of stimuli on sublimity. Brown noise was rated significantly higher on sublimity than white noise, pink noise, and voice recordings. Similarly, the combined voice recordings were rated significantly higher on sublimity compared to white noise and pink noise. There was also a significant difference between pink noise and white noise (see Table 4 for details).

**Table 4:** Wilcoxon signed-rank test, for sublimity ratings.

Emotion	Stimuli	Median	*z*	*N*	Sig (two-tailed)	*r*
Sublime	Brown noise- White noise	2 1	−16.64	1,277	<0.001	0.1
	Brown noise- Pink noise	2 1	−6.75	1,277	<0.001	0.1
	Brown noise- Voice recordings	2 1.5	−13.34	1,277	<0.001	0.3
	Voice recordings- White noise	1.5 1	−6.92	1,277	<0.001	0.1
	Voice recordings- Pink noise	1.5 1	−6.75	1,277	<0.001	0.1
	Pink noise- White noise	1 1	−12.77	1,277	<0.001	0.3

#### Unease

The results of a Friedman test indicated that there was a statistically significant difference in unease ratings for brown, pink, and white noise, and voice recordings *X*^2^ (3, *n* = 1,267) = 745.8, *p* < 0.001. A Wilcoxon signed rank test revealed a statistically significant difference between all six pairs of stimuli on unease. White noise was rated significantly higher on unease than brown noise, pink noise, and voice recordings. Similarly, pink noise was rated significantly higher on unease than brown noise and voice recordings. In addition, brown noise was rated significantly higher on unease compared to the combined voice recordings (see Table 5 for details).

**Table 5:** Wilcoxon signed-rank test, for unease ratings.

Emotion	Stimuli	Median	*z*	*N*	Sig (two-tailed)	*r*
Unease	White noise- Brown noise	5 3	−15.41	1,277	<0.001	0.4
	White noise- Pink noise	5 4	−6.13	1,277	<0.001	0.1
	White noise- Voice recordings	5 2.1	−23.49	1,277	<0.001	0.6
	Pink noise Brown noise	4 3	−14.25	1,277	<0.001	0.3
	Pink noise- Voice recordings	4 2.1	−20.51	1,277	<0.001	0.5
	Brown noise- Voice recordings	3 2.1	−10.61	1,277	<0.001	0.2

#### Vitality

The Friedman test results indicated a statistically significant difference in vitality ratings for brown, pink, and white noise, and voice recordings *X*^2^ (3, *n* = 1,267) = 122.9, *p* < 0.001. A Wilcoxon signed rank test revealed a statistically significant difference between five out of six pairs of stimuli on unease. Voice recordings were rated significantly higher on vitality than the pink noise. There was also a significant difference between pink noise, brown noise, and white noise (see Table 6 for details). For visual representation see Figure 3.

**Table 6:** Wilcoxon signed-rank test, for vitality ratings.

Emotion	Stimuli	Median	*z*	*N*	Sig (two-tailed)	*r*
Vitality	Voice recordings- Pink noise	1.3 1	−8.22	1,277	<0.001	0.2
	Pink noise- Brown noise	1 1	−9.46	1,277	<0.001	0.2
	Pink noise- White noise	1 1	−8.95	1,277	<0.001	0.2

**Figure 3:** Displays the three noises (brown, pink, and white) and the combined voice recordings and their respective median score for each second-order factor in the GEMS-9 scale. The error bars show the interquartile intervals (25th and 75th).

## Comparing studies 1 and 2

To compare studies 1 and 2 we did a Mann–Whitney U test, comparing the median scores on the emotional ratings for brown, pink, and white noise, as well as the combined voice recordings (see detailed results in Table 7). There was a significant difference between brown noise ratings of vitality in study 1 and study 2, as well as unease. There was a significant difference between pink noise ratings of vitality in study 1 and study 2, as well as unease. There was a significant difference between white noise ratings of uneasy in study 1 compared to study 2. There was a significant difference between voice recording ratings of sublimity in study 1 and study 2. See Figures 4–6 for visual representation of the respective second-order factors.

**Table 7:** Mann-Whitney U test comparing stimuli across Study 1 and Study 2 on sublimity, unease, and vitality ratings.

Group	*N*	Stimuli	Md	*U*	*z*	Sig.	*r*
Study 1	83	Brown noise vitality	1.5	45,970	−2.280	0.023	0.05
Study 2	1,273		1				
		Brown noise uneasy	1.5	33,940	−5.592	0.001	0.14
			3				
Study 1	83	Pink noise vitality	2	45,017	−2.477	0.013	0.06
Study 2	1,273		1				
		Pink noise uneasy	2	31,494	−6.249	0.001	0.16
			4				
Study 1	83	White noise uneasy	3	32,524	−5.991	0.001	0.16
Study 2	1,273		5				
Study 1	82	Voice recordings-sublimity	1.2	42,780	−2.694	0.007	0.07
Study 2	1,267		1.5				

**Figure 4:** Displays the significant differences in sublimity between study 1 (*N* = 84) and study 2 (*N* = 1,280). There was only a significant difference for the combined voice recordings measured with a Mann–Whitney U test. The figure shows the median values. The error bars show the interquartile intervals (25th and 75th).

**Figure 5:** Displays the significant differences in unease between study 1 (*N* = 84) and study 2 (*N* = 1,280). There was a significant difference for brown, pink, and white noise measured with a Mann–Whitney U test. The figure shows the median values. The error bars show the interquartile intervals (25th and 75th).

**Figure 6:** Displays the significant differences in vitalilty between study 1 (*N* = 84) and study 2 (*N* = 1,280). There was a significant difference for brown and pink noise measured with a Mann–Whitney U test. The figure shows the median values. The error bars show the interquartile intervals (25th and 75th).

## Discussion

The current two studies aimed to systematically evaluate the rating of emotion perceived in brown, pink, and white noise, as well as voice recordings, to explore to which degree these stimuli are suitable as control stimuli in studies on music perception.

Our first hypothesis was correct in both studies; white noise was rated as higher on unease compared to brown and pink noise, as well as voice recordings. However, it is important to note that the effect sizes, although above the required level by our G*Power calculations, were lower in Study 2, with effect sizes below the 0.5 level.

Our second hypothesis was partly rejected in both studies 1 and 2, as the noise stimuli did not indicate minimal emotional ratings for unease. While this only applied to white noise in study 1, it applied to brown, pink, and white noise in study 2. Brown noise was consistently rated as significantly more sublime compared to other noises in both studies but with low ratings. White noise was consistently rated higher for unease compared to the other stimuli. Pink noise, however, was consistently considered more vital than the other two noises, although with overall low ratings and effect sizes.

Unease ratings significantly increased in study 2 for all noises, however, the other emotions were not significantly different in studies 1 and 2. Another important observation is the variation in effect sizes across the studies. In study 1, all effect sizes were consistently moderate to large as defined by Cohen (1988). However, in Study 2, the effect sizes varied from small to large. This discrepancy between the studies might be due to what the noises and voice recording were compared to. Study 1 only consisted of voice recordings and noises, and the voice recordings intended as emotional stimuli did not get higher ratings than the assumed non-emotional stimuli. In Study 2, the non-emotional stimuli were compared to music. The differences in effect sizes might also be due to the sample size differences in the two studies, as effect sizes represent the magnitude between the groups (Sullivan and Feinn, 2012). With a larger sample size, it is natural that the groups are more different, and higher power as we had in study 2 also increases the chances that the statistically significant results represent a true effect (Button et al., 2013). In addition, Study 1 used the full GEMS-9, where participants could choose from nine different emotional words, rather than three in Study 2.

Our studies prompt crucial reflections on the appropriateness of using brown, pink, white noise and voice recordings as control stimuli in research settings. The use of brown, pink, and white noise aligns with Koelsch and Jäncke's (2015) recommendations for acoustical control stimuli in contrast with music and supports Chanda and Levitin’s (2013) suggestion for a non-musical control stimulus. However, it may not be ethically appropriate to use a stimulus that participants perceive as high in tension and unease. Although there is also some fluctuation between previous research and our current findings for brown, pink, and white noise.

For white noise, the findings from our studies align somewhat with prior research, where participants rated white noise as unpleasant (Bishop et al., 2009; Masuda et al., 2018). White noise has also been rated as giving significantly less joy and engagement and more sadness compared to music (Lynar et al., 2017). In addition, white noise increases anxiety for nursing students when played in the background during work conditions (Aksoy and Ozturk, 2024). Yet, it is hard to compare our study to others as we used different emotional wording; however, sadness and unpleasantness might be synonyms for unease. Regardless, our research and previous research indicate that white noise cannot be considered a “neutral” control stimuli, as it has been rated emotionally in several studies.

As for pink noise, it also indicated unease in Study 2. Intriguingly, a reduction in cognitive anxiety has been reported when participants listen to music, auditory beat stimulation, and pink noise compared to music and auditory beat stimulation combined (Mallik and Russo, 2022). This disparity in outcomes emphasizes the complexity of noise perception. However, it underscores the necessity for further research to understand pink noise.

Brown noise was rated consistently as more sublime than the other noises in both studies. This aligns with an earlier study (Voss and Clarke, 1978), suggesting that if we equate feelings of sublimity with pleasantness, brown noise was considered more pleasant than white noise. In a case study (Krasnoff and Chevalier, 2023), all four conditions -brown noise alone, brown noise and binaural beats, brown noise and music and brown noise, and music and binaural beats showed a relaxing brain, calculated by EEG readings in Alpha Assessment and CZ Theta Beta. Participants also had improved cardiovascular scores. Interestingly, the authors hypothesized that pink noise was more unpleasant than brown noise, therefore choosing not to use pink noise, which aligned with our findings from studies 1 and 2. We found that pink noise was rated significantly higher on unease compared to brown noise. Moreover, in study 2, brown noise was rated significantly more sublime than pink noise, although this distinction was not observed in study 1. Perhaps not surprisingly, music induces different patterns of activity in the prefrontal cortex, detected by near-infrared spectroscopy (NIRS) compared to brown noise (Moghimi et al., 2012). However, the authors used brown noise as a “neutral” control stimulus, while in our second study, we found that brown noise was rated with a median of 3 for unease in study 2. If we define neutrality as something with minimal emotional response (Gasper et al., 2021), then brown noise is not a neutral stimulus.

The voice recordings were created to elicit minimal emotional responses and be a neutral control stimulus. Some studies (Moghimi et al., 2012; Nyklíček et al., 1997; Russo et al., 2013) categorized noises as neutral conditions, leading us to question the definition of a neutral condition. In this study, we characterized a neutral stimulus as one that is rated with minimal emotional responses, which applied for brown and pink noise as well as voice recordings in study 1 and only voice recordings in study 2. Participants have reported feelings of neutrality alongside other feelings (Gasper et al., 2021) for stimuli, which is probably what we see in our studies. There was no option for no rating of emotion other than limiting responses to low numbers. Neutrality can be hard to assess, as participants tend to report positive responses when they do not have an opinion (Cacioppo et al., 1997). However, in our studies, the response was not positive but rather negative if we consider unease a negative feeling. We were successful in creating “neutral” voice recordings with minimal emotional response. Yet, the emotional voice recordings were not rated with strong emotional responses, so in that aspect. To create neutral stimuli, a much larger study with more stimuli and more participants is needed.

Other control stimuli that can be studied are, for example, natural environmental or animal sounds (Frühholz et al., 2016; Lepping et al., 2016). Some studies have used photographs of faces showing emotion to control for the emotional perception of music (Nawrot, 2003; Proverbio et al., 2015) as well. Furthermore, a picture database has been created to have tiers of univalence and neutrality for emotion research (Hahn et al., 2024). Using pictures is a different type of control stimuli, although it does not “match” auditory stimuli, which is why Koelsch and Jäncke (2015) do not recommend it for studies with music.

It would be beneficial for future studies to compare brown, pink, and white noise as well as voice recordings with silence, music, and other stimuli, considering both emotional and physiological parameters. There is also a need for more research on active or passive control conditions. Additionally, there needs to be a discussion on whether control stimuli should be neutral or if they should be as close to the variable we wish to test to obtain the most stringent results. We think it would be useful to have a meta-analysis or systematic review of the use of control stimuli in studies on music and emotion. Finaly, our findings hopefully contribute insight into the emotional perceptions associated with these noises and voice recordings, shedding light on their potential role as control conditions.

## Limitations

A limitation in our studies is the lack of control for sound levels in studies 1 and 2. Many prior investigations in white noise and pink noise have specified dB levels, highlighting the potential significance of this factor (Masuda et al., 2018). We could not control the decibel level as participants could adjust the volume themselves. Conducting surveys at home, as opposed to in a lab setting, introduces ecological validity (Honing and Ladinig, 2008; Pascoe et al., 2022). Addressing sound levels and performing headphone checks could enhance the robustness and consistency of future research.

There is a potential discrepancy between the translated Norwegian version of the GEMS-9 and the original English version, with some participants expressing concerns about the everyday application of the naturalness of the terms “sublimity,” “vitality,” and “unease” for emotional ratings. Notably, a study (Lykartsis et al., 2013) did an online survey testing the GEMS-9 scale in German and English, they found the German translation worked better than the original English version. Similarly, the GEMS-9 has been translated into Finnish (Eerola and Vuoskoski, 2011; Vuoskoski and Eerola, 2011), although no language bias was reported. More research is needed to understand the complexity of linguistic nuances and cultural considerations in the translation and application of emotion and music scales.

An additional problem with using the GEMS-9 is that it was meant for music and not control stimuli. We had to use the GEMS-9 because these studies were part of a larger project on music and emotion, which required consistency across all the studies.

## Conclusion

We found that noises were rated for specific emotions across two separate studies. The results raise critical considerations regarding the suitability of these noises to be used as control stimuli. Our studies also raised the question of what a neutral control stimulus is, and we have defined neutrality as low emotional ratings.

White noise had higher ratings for unease compared to brown and pink noise, as well as voice recordings in both studies. Only the combined voice recordings were considered neutral, defined as having consistently minimal emotional ratings in both studies.

Brown, pink, and white noise does not qualify as a “neutral” control condition due to its capacity to induce specific emotional responses, typically negative as uneasy, unpleasant, and sad. Furthermore, the existing literature appears to lack studies where these noises are systematically rated for emotion. This underscores the need for further exploration and evaluation of the emotional impact of brown, pink, and white noise. It is recommended for future studies to conduct and report a separate analysis for control conditions.

## Data Availability

The raw data supporting the conclusions of this article will be made available by the authors upon request.

## Footnotes

^1^ https://www.bksv.com/en/transducers/simulators/head-and-torso
